# Analysis of the Application Value of X-Ray Digital Tomographic Fusion Technique in Urinary System Diseases

**DOI:** 10.1155/2022/6294752

**Published:** 2022-01-07

**Authors:** Chensi Ouyang, Xiufang Yang, Jinghong Xie, Jinqiang Hu

**Affiliations:** ^1^Department of Urology Surgery, Yichun People's Hospital, Yichun 336000, Jiangxi, China; ^2^Radiology Department, Qingdao Eighth People's Hospital, Qingdao, Shandong 266100, China; ^3^Imaging Technology Department, Changle People's Hospital, Weifang, Shandong 262400, China

## Abstract

**Objective:**

To explore the application value of the X-ray digital tomographic fusion technique in the diagnosis of urinary system diseases.

**Methods:**

500 patients with suspected urinary diseases in our hospital were examined by three methods: X-ray digital tomographic fusion imaging (DTS), intravenous pyelography (IVP), and abdominal plain film (KUB), and the image quality before and after tomographic fusion was objectively evaluated. The image quality could be divided into three grades: excellent, good, and poor.

**Results:**

The image excellent rate of DTS (88%) was higher than that of IVP (27.5%). The sensitivity of DTS in the diagnosis of renal cyst and space occupying of the bladder was higher than that of IVP (*P* < 0.05). The accuracy rate of DTS in the diagnosis of urinary calculi was 93.33%, higher than 63.3% of KUB (*P* < 0.001). The accuracy rate of DTS in the diagnosis of ureteral stricture was 90%, higher than 65% of IVP (*P*=0.03). The accuracy of DTS in the diagnosis of hydronephrosis was higher than that of IVP and KUB (*P* < 0.05).

**Conclusion:**

In the examination of urinary system-related diseases, high-definition images can be obtained by timely using sectional fusion technology. Compared with conventional IVP, space occupying lesions such as the bladder and kidney can be displayed more clearly with the help of the tomographic fusion technique, which is helpful to improve the possibility of finding lesions and is of great significance in clinical application.

## 1. Introduction

In recent years, under the background of the rapid development of computer technology, a new imaging technology has gradually emerged, which is based on digital X-ray photography, that is, digital tomographic fusion imaging technology [1, 2]. The application of this technology not only has the advantages of low dose and high efficiency but also has the outstanding characteristics of high detection rate. Now, the clinical application of this technology has been gradually realized [3]. At present, intravenous pyelography is the most common method in the imaging examination of urinary diseases, but in the use of routine examination techniques, the results are often affected by many factors, such as low-density shadow and abdominal fat. This is not conducive to the accurate diagnosis of related diseases [4–6]. Therefore, it is very important to explore a scientific and accurate method for the diagnosis of urinary diseases. Some recent studies have found that through the application of digital tomographic fusion technology, the images of the above factors can be effectively avoided and high-definition images can be obtained. Find the focus in time [7, 8]. In this study, patients with urinary diseases treated in our hospital in the past half a year were included as the research subjects. After they were divided into groups according to different diagnostic methods, their clinical data were analyzed retrospectively. The purpose of this study is to explore the value of the X-ray digital tomography fusion technique in the diagnosis of urinary system diseases. The basic situation is reported as follows.

## 2. Materials and Methods

### 2.1. General Information

From September 2018 to February 2020, thousands of patients with abdominal and lumbar discomfort were treated in our hospital. Through direct contact and observation, these patients were suspected to have urinary tract diseases such as bladder or kidney space occupying. In this study, 500 patients with renal cyst, or space occupying of the bladder, or urinary calculi, or ureteral stricture, or hydronephrosis were selected, including 210 females and 290 males, all aged between 44 and 69 years old, with an average age of 59 years. The 500 patients were defined as the DTS group, in the examination process, the use of digital tomographic fusion technology assist in the diagnosis. All patients signed the informed consent. This study was approved by the Ethics committee of Changle People's Hospital.

### 2.2. Equipment and Method

In the process of examination of urinary diseases, two kinds of equipment are mainly used, the first is the image postprocessing workstation and the second is the Shimadzu multifunction large flat-panel digital photography system. In the process of specific examination, first of all, the doctor needs to guide the patient to lie flat on the examination bed in a supine position; second, take a plain film of the abdomen and protect the important organs of the patient that are not involved in the shooting. After that, routine IVP examination can be carried out. The specific steps are as follows: 40 milliliters of iohexol are injected intravenously into the patient, and the posterior abdomen is pressurized. Five minutes later, the renal calyx and renal pelvis are observed through fluoroscopy to determine whether they are full or not, and the films are taken at 7, 15, and 30 minutes, respectively. During this period, spot films are taken at an appropriate time according to the filling state of the ureter, renal calyx, and renal pelvis. When suspicious morphological and structural abnormalities are observed, it is necessary to use tomographic fusion imaging to examine the areas of interest. Specific steps are as follows: identify the key areas that need to be observed, adjust the center of the X-ray tube to aim at this area, and adjust the corresponding size of the aperture; the condition is 8 milliseconds, 85 kV. At 400 Ma, the detector and the tube move in a state of opposite parallel motion, with a total of 74 continuous exposures. When the relevant data are collected, all the relevant data need to be transmitted to the workstation, any 2 mm plane is reconstructed, and finally, the image of the continuous layer is obtained.

### 2.3. Image Observation and Analysis

Through the observation of the relevant images of this study, we analyzed the display effect of conventional VIP images and sectional fusion images, objectively compared the display ability of the two methods, found out the surrounding boundaries of space occupying lesions, measured them finely, and effectively evaluated the compression of the surrounding structures. According to the obtained image quality, refinement can be divided into three grades: excellent, good, and poor, that is, for KUB, if the psoas major muscle is very clear, the overall outline of the kidney is very clear, and the quality is excellent if it reaches the xiphoid process and down to the pubic symphysis. Meeting some of these 3 requirements is good; meeting only one requirement is poor. For the requirements of intravenous renography, if the outline of the kidney can be clearly seen, the development of the renal calyx and renal pelvis can be clearly seen, and all the images of the urinary tract can be clearly seen; if the outline of the kidney can be roughly identified and the development of the renal calyx and renal pelvis can be clearly seen, all the images of the urinary tract are relatively light. If the outline of the kidney is blurred, it is difficult to see clearly, the development of the whole urinary tract is blurred, or no development is defined as poor.

### 2.4. Statistical Method

The data were analyzed by SPSS 25.0 statistical software. The chi-square test was used to compare the counting data, and the rank sum test was used to compare the grade data. The difference was statistically significant (*P* < 0.05).

## 3. Results

Before the application of TDS, there were 2000 conventional KUB and IVP, of which 550 were excellent, 1100 were good, and 350 were poor. A total of 500 sectional fusion images were selected, including 440 excellent images, 60 good images, and 0 poor image (Table 1). All the selected patients completed the IVP examination successfully according to the plan. Through the observation and analysis of the images, it was found that there were 200 cases with abnormal bladder filling. Among the 200 patients, 140 cases had been confirmed to have bladder space occupying phenomenon, with the filling loss of bladder contrast agent as the specific manifestation, and the edge of the missing part showed irregular rules. The other 60 cases were suspected filling defects, which may have been affected by pelvic gas and intestinal contents. There were 60 patients who did not show abnormal bladder filling when the contrast medium was completely filled. There are 160 patients with renal cysts, with renal calyceal compression, deformation, and other phenomena, the edge of the renal pelvis is relatively smooth, and there are arc impressions. There are also 60 patients in the mode of complete filling of the contrast medium; affected by the lack of intestinal preparation, the gas produced greater interference, did not show the renal pelvis very clearly, and the structure of the renal calyx was abnormal. It was found that the renal pelvis and calyx of 20 patients developed very clearly and could easily distinguish the outline of the kidney. After DTS examination, renal cysts with small diameter were found around the renal parenchyma of the patients. During the routine IVP examination, the areas of interest were found, and the tomographic fusion scan was performed at the same time. A total of 250 cases of renal cysts were found, including 250 cases of bladder mass, 300 cases of calculi, 200 cases of ureteral stricture, and 260 cases of hydronephrosis. In this study, DTS combined with IVP and routine IVP were used. For renal cysts, the sensitivity was 100% vs. 72%, *P* < 0.05, and for bladder mass, the sensitivity was 100% vs. 64%, all *P* < 0.05 (Table 2). The diagnostic accuracy of DTS and KUB for urinary calculi was 93.33% vs. 63.3%, *P* < 0.05 (Table 3). Using DTS and IVP, respectively, the diagnostic accuracy of ureteral stricture was 90% vs. 65%, *P* < 0.05 (Table 4). DTS was used for the diagnosis of hydronephrosis, and the detection rate of IVP and KUB was compared with 92.3% vs. 65%, *P* < 0.05 (Table 5). In the process of scanning using sectional fusion technology, all images successfully avoid the influence and interference of intestinal volume and intestinal gas.

## 4. Discussion

In the X-ray traversing track, a variety of arbitrary number of target layers can be formed during the tomographic fusion imaging examination. The X-ray can carry out continuous projection in the process of moving through multiple angles [9–11]. Compared with the direction of the patient's movement, the detector and the stadium move at the same time and are balanced and opposite to the patient's movement [12, 13]. Then, a number of related projection images can be collected quickly, and then, the collected images can be reconstructed with the help of the SAA program, and the cross-sectional images with any set height can be reconstructed successfully under the operation of the program [14, 15].

At this stage, in the examination of urinary diseases, including kidney stones, hydronephrosis, and other diseases, the use of conventional IVP still plays a very important role and still has its application value in the examination of urinary tract diseases [16]. In this study, the one-time imaging of IVP and DTS is organically combined. After proper processing and arrangement, the focus can be revealed more clearly by observing and analyzing the sectional images of key parts [17, 18]. In this study, after the application of tomographic fusion technology, the image of the patient's renal pelvis is very clear, but only using conventional intravenous renography, the renal calyx and renal pelvis are relatively blurred. Moreover, the development of some patients is relatively poor, and it is even difficult to show the development. The reason is mainly due to the interference of the gas in the gastrointestinal tract of the patients, as well as the influence of the contents. For the patients who were diagnosed as bladder space occupying in this examination and were suspected to be bladder cancer, the image in which the contrast medium had been very full after waiting for 30 minutes was observed. It is found that the position of bladder space cannot be accurately determined by this image, let alone the size of its range; while, tomographic fusion imaging can avoid all kinds of interference, and the size and position of bladder space can be found quickly and clearly by observing the image. In the link of this abdominal examination, it is found that compared with ordinary examination, tomographic fusion imaging can also improve the detection rate of stones. Ordinary examination will not only be disturbed by intestinal contents but also be affected by gas. Stones with smaller shape and lower density cannot be displayed, but through tomographic fusion imaging, stones with small shape and low density can be clearly displayed. 15 minutes after the injection of the contrast medium into a patient, the routine examination showed that the right renal pelvis was very clear, and the renal calyx was also clearly developed, but due to compression, the left renal pelvis and calyx formed an arc. The patient was diagnosed as a left renal cyst; through the sectional fusion image, the size, scope, and location of the patient's left renal cyst can be clearly found, and the edge of the cyst can also be clearly seen. When the contrast medium was injected into the patient with left renal cyst, the image taken by routine examination 15 minutes later was not clear because the patient's gastrointestinal tract was not prepared, and there was too much content and intestinal gas. The left and right renal pelvis and calyx are not clearly shown.

The application of digital tomographic fusion technology can effectively solve the overlap problems encountered in conventional IVP examination, successfully avoid the interference caused by intestinal fecal shadow, and play a positive role in improving the display rate of urinary system diseases. In this selection of 500 patients with urinary diseases, the application of the tomographic fusion technique has a very high clinical diagnostic value for patients with inadequate intestinal preparation, and the lesions are relatively small and not obvious. For example, when a patient is diagnosed with a renal cyst, the renal pelvis has been caused, and the overall outline of the renal calyx has changed to a certain extent, if the conventional intravenous renography is used, it is difficult to clearly show the outline of the renal calyx and other parts of the kidney. The use of sectional fusion technology can effectively solve this problem, which is of great practical significance for the diagnosis of renal cysts, regardless of the size of the cyst. Or the location and scope can be clearly seen by the doctor. Therefore, in the examination of urinary diseases, although intravenous renography has been widely used in clinics and has certain practical significance, the timely use of the tomographic fusion technique can more effectively and clearly observe the real situation of related body parts such as the ureter, bladder, and kidney, as long as we find the best time to take pictures for patients, so as to further improve the speed of radiography. And the interference of overlapping intestinal contents and gases can also be effectively avoided, so as to effectively measure the size, location, and extent of the lesions.

X-ray wavelength is relatively short, probably between 0.01 and 10 mm, has a good penetration performance, and human beings cannot be observed with the naked eye [18, 19]. Different from other rays, because X-ray has very strong characteristics in diagnosis, it can be widely used in many fields of medicine, and it has been used earlier in medical imaging [20]. When passing through the material of different densities, the penetration ability of X-ray is also different, and in the process of transmission, the energy produced is continuously absorbed by the material. The output voltage is the decisive factor affecting the penetration ability of X-ray; if the voltage given to it is weak, then the penetration ability of X-ray will be weak; if it is given a higher voltage, then the penetration ability of X-ray will be relatively strong [10]. According to the principle of X-ray imaging, in the process of irradiation, photosensitivity and fluorescence effects are gradually formed according to the basis of imaging. When the human body is irradiated by X-ray, the imaging is formed according to the imaging after irradiation. At the same time, it is produced by combining with the internal structure of the human body. In the same tissue, the different places of imaging are found to be the so-called pathological changes [21].

In the examination of urinary diseases, as a routine examination method, such as KUB and IVP, it has been widely used in clinics [22]. The examination method of KUB has the advantage of simple and easy; in urinary diseases, most of the positive stones can be diagnosed effectively and accurately, and the application of intravenous pyelography can observe the site of urinary tract obstruction. It is of practical significance for the diagnosis of renal parenchyma tumors [7, 23]. Although the above two routine examination methods have their own advantages and play a very important role in the diagnosis of urinary diseases, they may be affected by overlapping images of intestinal contents and intestinal gases of the patients. As a result, the image of the anatomical structure of the urinary system is not clear enough, the location of the lesion cannot be accurately displayed, and it is difficult to achieve the diagnostic goal [24]. The use of digital tomographic fusion technology is to use a receiver, and it is fixed; through the use of single-layer imaging scanning, a series of exposure images are collected in this process, and the collected data are reconstructed scientifically, and then, start from the surface of the receiver to the imaging anatomy, and the multiple planes involved are displayed [25, 26]. In this way, not only the shape and outline of the kidney and ureter in the urinary system can be shown clearly but also the more subtle structure of the renal pelvis and calyx can be clearly displayed, and the edge shape of the focus can be shown more clearly, as well as the subtle changes of the adjacent structure, which can greatly improve the clarity and contrast of the urinary system image.

To sum up, in the examination of urinary diseases, compared with the commonly used methods such as KUB and IVP at the present stage, as a new method of clinical diagnosis, the application of the DTS technique can improve the success rate of initial examination of related diseases without intestinal preparation and can effectively avoid the interference of gas, intestinal contents, and other factors in the field. The size and range of lesions can be measured efficiently, which plays an important role in clinical diagnosis.

## Figures and Tables

**Table 1:** Comparison of the excellence rate of DTS inspection and IVP inspection images.

	Excellent	Good	Poor	Total	Excellence rate (%)
DTS	440	60	0	500	88
IVP	550	110	350	2000	27.5

**Table 2:** Comparison of sensitivity between DTS and IVP in renal cyst and bladder space occupying lesion.

	DTS	IVP
Renal cyst (*n* = 250)	240	180
Bladder space occupying lesion (*n* = 250)	250	160
	*P* < 0.001	

**Table 3:** Comparison of the accuracy of DTS and KUB in the diagnosis of urinary calculi.

Method	*n*	Accurate	Inaccurate	Accuracy rate (%)
DTS	300	280	20	93.33
KUB	300	190	110	63.3
	*P* < 0.001			

**Table 4:** Comparison of the accuracy of DTS and IVP in the diagnosis of ureteral stricture.

Method	*n*	Accurate	Inaccurate	Accuracy rate (%)
DTS	200	180	20	90
IVP	200	130	70	65
	*P*=0.03			

**Table 5:** Comparison of the accuracy of DTS, IVP, and KUB in the diagnosis of hydronephrosis.

Method	*n*	Accurate	Inaccurate	Accuracy rate (%)
DTS	260	240	20	92.3
IVP or KUB	260	170	90	65.4
	*P* < 0.001			

## Data Availability

The analyzed datasets generated during the study are available from the corresponding author upon request.
